The article "The Impact of the Declaration of the State of Emergency on the Spread of COVID-19: A Modeling Analysis" was published in 2021. Journal: Comput Math Methods Med.

# The Impact of the Declaration of the State of Emergency on the Spread of COVID-19: A Modeling Analysis

**DOI:** 10.1155/2021/8873059

**Published:** 2021-07-26

**Authors:** Zhongxiang Chen, Siqiang Sun, Wenhui Zhao, Zhaoru Liu, Xinyao Zhao, Xiuxiang Huang, Jiaji Pan

**Affiliations:** ^1^College of Engineering and Design, Hunan Normal University, Changsha, Hunan, China 410081; ^2^State Key Laboratory of Developmental Biology of Freshwater Fish, Hunan Normal University, Changsha, Hunan, China 410081

## Abstract

When encountering the outbreak and early spreading of COVID-19, the Government of Japan imposed gradually upgraded restriction policies and declared the state of emergency in April 2020 for the first time. To evaluate the efficacy of the countering strategies in different periods, we constructed a SEIADR (susceptible-exposed-infected-asymptomatic-documented-recovered) model to simulate the cases and determined corresponding spreading coefficients. The effective reproduction number *R*_*t*_ was obtained to evaluate the measures controlling the COVID-19 conducted by the Government of Japan during different stages. It was found that the strict containing strategies during the state of emergency period drastically inhibit the COVID-19 trend. *R*_*t*_ was decreased to 1.1123 and 0.8911 in stages 4 and 5 (a state of emergency in April and May 2020) from 3.5736, 2.0126, 3.0672 in the previous three stages when the containing strategies were weak. The state of emergency was declared again in view of the second wave of massive infections in January 2021. We estimated the cumulative infected cases and additional days to contain the COVID-19 transmission for the second state of emergency using this model. *R*_*t*_ was 1.028 which illustrated that the strategies were less effective than the previous state of emergency. Finally, the overall infected population was predicted using combined isolation and testing intensity; the effectiveness and the expected peak time were evaluated. If using the optimized control strategies in the current stage, the spread of COVID-19 in Japan could be controlled within 30 days. The total confirmed cases should reduce to less than 4.2 × 10^5^ by April 2021. This model study suggested stricter isolating measures may be required to shorten the period of the state of emergency.

## 1. Introduction

The coronavirus disease (COVID-19) caused by severe acute respiratory syndrome coronavirus (SARS-CoV-2) has been spreading since the first case report in December 2019 [1, 2]. By May 16, 2021, the COVID-19 confirmed cases reached over 160 million cumulatively with a reported 3.3million deaths [3].

To curb the spread of this pandemic, strategies were imposed by policymakers in various countries such as school closure, suspension of public events, restricting travelling from early infected countries, self-isolation orders, large-scale quarantine, and strict lockdown measures [4–6]. However, the strict measures brought great socioeconomic pressure [7]. Most countries may lack a political will or the ability to persist with extreme strict containment policies [8]. The COVID-19 containing strategy could be adjusted and optimized to be implemented in different countries. The first case in Japan was confirmed on Jan 15, 2020. The government proposed a basic control policy on February 25, 2020, and revised the policy on March 28, 2020. Due to the worsening situation, 3817 infected cases were confirmed, the transmission route of over 40% of cases could not be tracked, and the government put forward a stricter control policy nationwide and declared a state of emergency. On May 25, 2020, the state of emergency was lifted after the daily confirmed cases reduced to less than 50.

The article "The Impact of the Declaration of the State of Emergency on the Spread of COVID-19: A Modeling Analysis" was published in 2021. Journal: Comput Math Methods Med.

The accumulated infected cases of COVID-19 reached 404472 as of Feb 08, 2021 in Japan [9]. After December 2020, a large number of COVID infections appeared, and the state of emergency was declared again in January 2021. The effect of the state of emergency could be analyzed in the approach by mathematical modeling. In the previous study, the effectiveness of the early strategies adopted by the Government of Japan was assessed using a susceptible-infected-removed- (SIR-) based stochastic transmission model [5]. The amount of time spent in the crowded zone should be reduced, but the feasibility of testing and isolation strategy was not emphasized in the model. Moreover, control strategies during different periods had been adopted, thus changed the disease transmission capacity. Therefore, it is difficult to accurately estimate the parameter values of the epidemic model. Kuniya [10] estimated the transmission rate coefficients based on a simple susceptible-exposed-infected-recovered (SEIR) model without considering the transmission rate from exposed individuals and the early imported cases. Since the proportion of asymptomatic people during the confirmed patients may be significant, the infectiousness of asymptomatic people should be considered as a nonnegligible source.

In many other studies, the mechanism analysis and evaluation of containing strategies were also applied. There is much work on the mechanism analysis and development prediction of COVID-19 using the traditional SEIR model [11–14]. However, some of these works ignore the infectivity of the incubation period (the time between the exposure of the virus and the appearance of the symptom). Infectivity in the latent period was considered by Jiao [11], implying that the governments should strictly implement the isolation system to curb the disease propagation. A dynamic epidemic model for COVID-19 was established considering infectivity in the incubation period and divided the population into three types of age groups. The results show that population-wide testing and contact tracing can effectively reduce the spread of disease. The environmental conditions were considered in [15], the SEIRV model is constructed, and *V* denotes the concentration of COVID-19 in the environmental reservoir. Their results indicate that the COVID-19 would remain endemic, which necessitates long-term disease prevention and intervention programs.

The article "The Impact of the Declaration of the State of Emergency on the Spread of COVID-19: A Modeling Analysis" was published in 2021. Journal: Comput Math Methods Med.

This study considered the influence of isolation measures, PCR test medical screening [16], and the infection by the asymptomatic cases [17]. We established a susceptible-exposed-infected-asymptomatic-documented-recovered (SEIADR) epidemic system. Specifically, we considered the compartment for analyzing the asymptomatic transmission due to the reported asymptomatic infections [18, 19]. In the SEIADR model, the influence of isolation and testing intensity was quantitively defined. The COVID-19 spreading period was partitioned into multiple stages primarily based on different essential basic policies put forward to control the pandemic. The parameter values of each stage were obtained by solving the optimization problem and fitting the real number of confirmed cases. In particular, the reduced transmission rates and effective reproduction number demonstrated the conductive effect of entering a “state of emergency” in the early stages. Adopting the established model, we analyzed the current situation in Japan in another state of emergency. Further, a number of combined strategies were simulated using this model to offer some guidance in containing the pandemic in Japan.

## 2. Methods

### 2.1. Model Description

We established the following SEIADR compartmental model to study the previous spreading of COVID-19 in Japan, characterize the current situation, and estimate the future development (Figure 1). According to the infectious characteristics of COVID-19, the facts that the exposed people during the latent period and asymtopmatic patients are infectious were taken into consideration in this epidemic model. The parameters in the model were adopted to characterize specific parts of the COVID-19 transmission and evaluate the severity of the pandemic in different stages. The structure of this SEIADR dynamic model was consistent with the dynamics of the disease spreading.

The epidemic system is characterized with the following equations:

(1) $$\begin{array}{c} \left\{\begin{array}{c} \dot{S}=-\beta_{e}SE-\beta_{i}SI-\beta_{a}SA,\\ \dot{E}=\beta_{e}SE+\beta_{i}SI+\beta_{a}SA-\mu E,\\ \dot{I}=\alpha \mu E-\gamma I,\\ \dot{A}=\left(1-\alpha \right)\mu E-\delta A-\varepsilon A,\\ \dot{D}=\delta A+\gamma I-\lambda D,\\ \dot{R}=\varepsilon A+\lambda D, \end{array}\right. \end{array}$$

where *S*, *E*, *I*, *A*, *D*, and *R* denote the susceptible, exposed (incubation period), infected, asymptomatic, documented, and recovered portion in the total populations, respectively. *S* compartment represents the susceptible cases. *E* compartment indicates the symptomatic cases who already got infected before the onset of symptoms. *I* compartment denotes infected cases who already got symptoms. *A* compartment represents asymptomatic cases that are infected without any symptoms. *D* compartment indicates the documented cases that have been isolated or quarantined. We assume these cases could not spread the disease. *R* compartment denotes the recovered cases. The number of confirmed cases including quarantined cases, cured cases, and death cases can represent the epidemic state of COVID-19. *β*_*e*_, *β*_*i*_, and *β*_*a*_ (per day) denote the transmission rate coefficients from the exposed (incubation period), infected (symptomatic), and asymptomatic patients, respectively. *μ* (per day) is the rate from the incubation period to the infected symptomatic individuals. The average incubation period is 1/*μ*. *α*represents the proportion of the infected patients with symptoms, and 1 − *α* represents the proportion of patients without symptoms. *γ* is the confirmation rate of symptomatic cases, and 1/*γ* is the average confirmation time. *δ* is the confirmation rate of the asymptomatic infections. The asymptomatic patients could only be screened and diagnosed by testing. (per day) is the recovery rate of asymptomatic infections, and *λ* (per day) is the recovery rate of confirmed infections. The average recovery time is 1/*ε* and 1/*λ*, respectively. The average recovery time for symptomatic infected and asymptomatic patients is set to be 21 and 14 days, respectively.

The article "The Impact of the Declaration of the State of Emergency on the Spread of COVID-19: A Modeling Analysis" was published in 2021. Journal: Comput Math Methods Med.

We assume that the confirmed cases will be quarantined without infectivity. The effective reproduction number *R*_*t*_ is derived following the procedure as described by Driessche and Watmough [20], and the matrix of the rate of new infections of the system (1) *ℱ* can be expressed as

(2) $$\begin{array}{c} F=\left[\begin{array}{ccc} \beta_{e}N_{0} & \beta_{i}N_{0} & \beta_{a}N_{0}\\ 0 & 0 & 0\\ 0 & 0 & 0 \end{array}\right]. \end{array}$$

The matrix of the rate of transfer of individuals of the system (1) *𝒱* can be expressed as

(3) $$\begin{array}{c} V=\left[\begin{array}{ccc} \mu & 0 & 0\\ -\alpha \mu & \gamma & 0\\ -\left(1-\alpha \right)\mu & 0 & \delta +\varepsilon \end{array}\right]. \end{array}$$

*R*_*t*_ is achieved as the spectral radius of the matrix *ℱ𝒱*^−1^ [20]:

(4) $$\begin{array}{c} R_{t}=\frac{\beta_{e}}{\mu }+\frac{\beta_{i}\alpha }{\gamma }+\frac{\beta_{a}\left(1-\alpha \right)}{\delta +\varepsilon }. \end{array}$$

### 2.2. Fitting of the Parameters

The least-square method is used to calculate the value of the parameters. For given parameters *β*_*e*_, *β*_*i*_, *β*_*a*_,*α*,*δ*, and *γ*, the accumulated confirmed cases by numerical simulation $\tilde{Y}\left(t\right)$ for a time range [*t*_0_, *t*_*L*_] are

(5) $$\begin{array}{c} \tilde{Y}\left(t\right)=\overset{t_{L}}{\underset{\tau =t_{0}}{\sum }}\left(\delta A\left(\tau \right)+\gamma I\left(\tau \right)\right), \end{array}$$

where *τ* represents a day during the period [*t*_0_, *t*_*L*_].

Let *Y*(*t*) be the real reported confirmed cases, and the following target function is set up:

(6) $$\begin{array}{c} J\left(\beta_{e},\beta_{i},\beta_{a},\alpha ,\delta ,\gamma \right)=\overset{t_{L}}{\underset{t_{0}}{\sum }}{\left[Y\left(t\right)-\tilde{Y}\left(t\right)\right]}^{2}, \end{array}$$

(7) $$\begin{array}{c} 0<\beta_{e},\beta_{i},\beta_{a},\alpha ,\delta ,\gamma <1. \end{array}$$

Thus, the determination of *β*_*e*_, *β*_*i*_, *β*_*a*_,*α*,*δ*, and *γ* should be converted into optimizing the target function:

(8) $$\begin{array}{c} \min J\left(\beta_{e},\beta_{i},\beta_{a},\alpha ,\delta ,\gamma \right). \end{array}$$

For a given time range [*t*_0_, *t*_*L*_], the initial value was set to be the state at *t*_0_ − 1 (*S*(*t*_0_ − 1), *E*(*t*_0_ − 1), *I*(*t*_0_ − 1), *A*(*t*_0_ − 1), *D*(*t*_0_ − 1),*R*(*t*_0_ − 1)). Upon the outbreak of the COVID-19, the initial value was set to be (*N*_0_, 1, 0, 0, 0, 0). The parameters were set in the range which all satisfied (7). The target function (6) was solved by a nonlinear least-squares fitting method using function lsqnonlin in MATLAB (built-in trust-region-reflective algorithm [21, 22]).

### 2.3. Data and Transmitting Stages in Japan

The data for the modeling analysis are collected from various sources including Japan's public broadcaster NHK, local government, and the organization of Our World in Data [23–25]. According to the public counter released from the Ministry of Health, Labour, and Welfare [26], the basic policy to contain the spread of COVID-19 was announced on Feb 24, 2020, and revised on March 25, 2020. Seven prefectures declared a state of emergency on April 6 2020. Nine days later, the state of emergency was extended to the entire Japan. The government put forward a stricter control policy nationwide and declared a state of emergency. On May 25, the state of emergency was lifted. On Jan 7, 2021, the Government of Japan declared a state of emergency again. We divided the time frame into different stages primarily according to the policy announced by the Government of Japan [3, 26–34] as shown in Table 1.

The article "The Impact of the Declaration of the State of Emergency on the Spread of COVID-19: A Modeling Analysis" was published in 2021. Journal: Comput Math Methods Med.

### 2.4. Fitting Transmission Parameters with Isolation Intensity and Testing Indexes

The transmission rate coefficients *β*_*e*_, *β*_*i*_, and *β*_*a*_ are inherently related to isolation and testing intensities. We consider using the average rate of increase of untraceable cases *p* to represent the isolation intensity. The daily numbers of untraceable cases since April 2020 are disclosed by the government [24]. The daily rate of increase of the untraceable cases is the number of untraceable cases compared with the data one week before, which is also released simultaneously. In each stage as divided in Table 1, we summed up the daily rate of increase of the untraceable cases and divided by the number of days at that stage. Hence, the average rate of increase of untraceable cases *p* for the stages was achieved, and the influence of different durations of stages could be eliminated. It is assumed that with a better isolation level, there should be fewer untraceable cases. We define the testing index *χ* as the testing numbers during each stage divided by the number of increased confirmation cases and the number of days at that stage. The testing index represents the average testing intensity for each stage which also avoids the influence of different durations of stages (Figure 2).

The transmission parameters *β*_*e*_, *β*_*i*_, and *β*_*a*_ are nonnegative. After taking the logarithms of the transmission parameters, we adopted exponential functions to fit the log-transformed parameters with the average rate of increase of untraceable cases *p* and average testing intensity *χ* by using the Curve Fitting app in MATLAB.

## 3. Results

### 3.1. Simulation Results and Associated Parameters in Different Stages

Based on the established SEIADR model, we conducted the simulation of the confirmed cases and achieved the parameters by fitting the case number and the model prediction curve. The portion of asymptomatic cases varies significantly according to different studies [35]. Simulated by this epidemic system, the asymptomatic percentage ranges from 66% to 88% (Table 2). As can be seen in Figure 3(a), the simulation curves generated by the model fit well with the reported confirmed cases. The simulated transmission and confirmation rates are shown in Table 2. The simulation of the accumulated confirmed cases is plotted with a 95% credible interval using the determined parameters (Figure 3(b)).

The article "The Impact of the Declaration of the State of Emergency on the Spread of COVID-19: A Modeling Analysis" was published in 2021. Journal: Comput Math Methods Med.

In the early spreading period, the transmission rate coefficients of the exposed *β*_*e*_, infected *β*_*i*_, and asymptomatic cases *β*_*a*_ are 0.1984, 0.5469, and 0.5094 (stage 1); 0.0803, 0.2454, and 0.2182 (stage 2); 0.3093, 0.6767, and 0.7014 (stage 3). As can be seen from the transmission coefficients, the spreading of COVID-19 was not well suppressed; although, several measures had been proposed in the early stages. The official encouragement to stay away from crowded places and promote teleworking to enhance social distancing may not be that effective, but the parameters representing the confirmation rates of symptomatic infected *δ* and asymptomatic *γ* by testing and increased in stage 3 suggesting more cases were determined and documented. Upon the declaring the state of emergency for several prefectures in stage 4 and expanded nationwide in stage 5, the transmission coefficient decreased to 0.0131, 0.4395, and 0.3264 (stage 4) and 0.0121, 0.2553, and 0.1869 (stage 5).

The effective reproduction numbers *R*_*t*_ determined in the first three stages are 3.5736 (95% CI [3.1484 4.5201]), 2.0126 (95% CI [1.5327 2.6484]), and 3.0672 (95% CI [2.6683 3.6140]). During the state of emergency in stage 4 and stage 5, *R*_*t*_ reduced to 1.1123 (95% CI [0.9464 2.3929]) and 0.8911 (95% CI [0.4197 1.923]), respectively. The spreading of infected cases was well controlled. The previous analysis illustrated COVID-19 infection spread in Japan could be inhibited by reducing the time spent in the public area and follow the basic policies in stage 2 [5]. However, those control strategies in that stage failed to prevent the further deterioration of disease spreading. The rapid spreading was controlled with more strict policies proposed in stage 4 and stage 5. The restrictions imposed by the authorities during the state of emergency were effective to inhibit the massive increment of infected cases.

After the lifting of the emergency state, the COVID-19 infections in Japan remain continuously growing with *R*_*t*_ 1.6312 (95% CI [0.1741 1.9746]). More recently, the second wave of massive infections occurred. On Jan. 7, 2021, the Japanese government declared the “state of emergency” again in view of the urgent need to increase the containing strategies. The transmission parameters are reduced to 0.0914, 0.4529, and 0.2674 (stage13). It was worth note that although in this period, the state of emergency was declared similarly as that was done in stage 5. The transmission rate coefficients are much larger than those in stage 5 (655% increase in *β*_*e*_, 77% increase in *β*_*i*_, and 43% increase in *β*_*a*_) which represents less effective control of the COVID-19 spreading in the nationwide state of emergency for the second time. It should result from different containing measures or increased infectivity of the virus [36]. The confirmation rates increased to 0.57 and 0.48, illustrating the strengthening testing strategies. After the second declaring state of emergency, *R*_*t*_ was reduced to 1.028.

The article "The Impact of the Declaration of the State of Emergency on the Spread of COVID-19: A Modeling Analysis" was published in 2021. Journal: Comput Math Methods Med.

### 3.2. Fitting Results of Parameters

By fitting the transmission rate coefficients *β*_*e*_, *β*_*i*_, and *β*_*a*_ with untraceable growth rate *p*, testing intensities *χ*, and the asymptomatic confirmation rate *γ*, we achieved the following relationships:

(9) $$\begin{array}{c} \beta_{e}=e^{-9.2839+11.901p-4.2453p^{2}-0.2638\chi -1.6474\gamma },\\ \beta_{i}=e^{-2.8451+3.4741p-1.2845p^{2}-0.032308\chi -0.37442\gamma },\\ \beta_{a}=e^{-2.6304+3.5011p-1.1832p^{2}-0.13608\chi -1.9964\gamma }. \end{array}$$

The coefficient of determination *R*^2^ [37] for these multiple regressions is 0.935, 0.985, and 0.908, respectively. The asymptomatic cases are more difficult to be detected compared to the symptomatic infected cases, which should pose more threat to the controlling of the COVID-19 spreading. By using the same method for the fitting of transmission parameters, the relationship between confirmation parameters *δ*, *γ*, and the testing index *χ* is achieved (plotted in Figure 4) as the following expression with *R*^2^ = 0.981:

(10) $$\begin{array}{c} \delta =\frac{1}{1+e^{1.502-1.16\chi -2.145\gamma }}. \end{array}$$

The confirmation rate represents the percentage of discovered asymptomatic cases and estimated existed asymptomatic cases. As can be found by fitting the testing index and the confirmation rate in the early six stages, the efficiency to determine asymptomatic cases by testing rapidly grows for smaller indexes. As the testing index increases, the confirmation rate tends to increase slower. Thus, it illustrates that it may of interest to avoid drastically increase the testing numbers. There should exists a bottleneck effect on the control of COVID-19 by increasing the testing intensity.

### 3.3. Accumulated Cases Trend with Combined Testing and Isolation Strategies

The simulated curve fits well with the real cumulative case reports as presented. Thus, the model was used to predict the future cumulative cases with the current containing policy as well as several modified strategies (Figure 5). The growth rate *p* and testing index *χ* for the current state of emergency are 1.1141 and 0.6016, respectively. If the isolation and testing intensities remain, the accumulated number of cases will continue to grow and reach 4.78 × 10^5^ in May 2021 based on the prediction (blue line in Figure 5(a)). In the scenario keeping the current testing index *χ* 0.6016, but increasing isolation intensity, corresponding to a smaller *p* value, the final number of infected cases will gradually reduce to less than 4.2 × 10^5^. More importantly, the growing trend of accumulated infected cases will slow down and reach a stable peak much faster. Increasing *p* to 0.6021, which is the same in stage 5 (the first nationwide declaration of a state of emergency) by taking the intensive isolation measure, the second wave of massive infections should be controlled by the end of February.

The article "The Impact of the Declaration of the State of Emergency on the Spread of COVID-19: A Modeling Analysis" was published in 2021. Journal: Comput Math Methods Med.

If keeping the same isolation intensity, increasing the testing index from 0.6016 to 1.6 instead, the time needed to control the COVID-19 spreading should not be significantly reduced. The accumulated confirmed cases decreased by 1.6 × 10^4^ by increasing *χ* from 0.6016 to 1.0. Further increasing *χ* from 1.0 to 1.4 could result in around 1 × 10^4^ less infected cases. The effect of increasing testing intensity should be revealed by the reduction in the accumulated confirmed cases. But for each varying testing intensity (Figures 5(a)–5(f)), the higher *p* value demonstrates dominance in shortening the time to get through rapid transmission period and reach the peak of accumulated cases.

The peak time contour map (Figure 6(a)) is plotted to determine the expected lasting days for different strategies with combination of testing index *χ* and untraceable growth rate *p* to reach a desired outcome. When *p* is higher such as larger than 1, corresponding to less strict isolating measures, it could reduce the peak time substantially by greatly increasing the testing index. If *p* declines down to less than 0.8 with implementing more strict isolation strategies, the effect of larger testing index should be insignificant. For the current stage, taking isolating strategies reducing *p* down less than 0.65 could end the state of emergency within 35 days with the current testing intensity.

Also, the effective reproduction number *R*_*t*_ is determined with the combination of various strategies (Figure 6(b)). It is suggested to control the pandemic transmission, and the strategy of combined isolation and testing intensity should locate in the lower right area of the green line so that *R*_*t*_ is less than 1.

### 3.4. Validation of the Prediction by the Model

The previous analysis and data fitting were performed from the outbreak of COVID-19 in Japan to Jan 27, 2021. To validate the model, we predicted infected cases during the period from Jan 28, 2021 to Feb 4, 2021 using the model parameters extracted from stage 13 during which the state of emergency is declared again (Figure 7). The real accumulated confirmed cases during that week locate in the 95% credible interval of simulated results. Together with the previous fitting and validation of the early transmission stages (Figure 3), the reliability of this SEIADR model is further strengthened after checking the current period. Controlling the second wave of massive infections should last longer than the first state of emergency if maintaining the isolation intensities in the current stage.

The article "The Impact of the Declaration of the State of Emergency on the Spread of COVID-19: A Modeling Analysis" was published in 2021. Journal: Comput Math Methods Med.

The parameters of the model used for prediction are extracted by the fitting the last stage between Jan 8, 2021 and Jan 27, 2021. The real number of confirmed cases falls within the 95% CI of the forecasted number during the period between Jan 28, 2021 and Feb 4, 2021.

## 4. Discussion

In this study, we developed a SEIADR mathematical model to simulate and analyze the development of COVID-19 epidemic in Japan. The transmission of the disease was divided into different periods. The modeling fitting and extraction of corresponding parameters were conducted for each specific stages. For the early COVID-19 transmission in Japan, we determined different stages based on the released policies by the government. After suppressing the first wave of a large number of infections in May 2020, the basic policies were not updated. The following stages were divided according to the modified partial strategies announced by the government. Since many hidden variables such as the personal willing to insist with the guidance and the infectibility may hardly be quantified, we employed a model with more compartments and adopted five parameters to fit the model with the real cases. The three transmission rate coefficients and two confirmation parameters inherently illustrate the overall effects of the containing strategies including isolation and testing intensities. After achieving these parameters, this study used two reported variables to perform a quantitative analysis. The two variables are correlated to the isolation effects and testing intensities by fitting with the transmission and confirmation parameters obtained from the model.

Compared to other models which are composed of three or four compartments [5, 11, 18], this study adopted six compartments to simulate the realistic transmission scenario. The infectiousness in the incubation period and the transmission resulted from the asymptomatic patients are taken into consideration. Differentiating the time into several stages ensures fitting the parameters dynamically, otherwise leading to misleading results. This analysis presents a more complex but more solid approach of analyzing the COVID-19 transmission in Japan.

The article "The Impact of the Declaration of the State of Emergency on the Spread of COVID-19: A Modeling Analysis" was published in 2021. Journal: Comput Math Methods Med.

The declaration of the state of emergency has played a significant role in controlling the disease as previously studied, either for the regional area [38] or expanded to entire Japan for the first time. Though, it was suggested by previous qualitative study suggested that Japan should implement more testing and mitigation measures during the first state of emergency [39]. Another study listed several unique measures in Japan to explain why Japan could enforce a loose restriction without large the collapse of medical resources or high fatality rate. This model demonstrates the effectiveness of the first declaration of a state of emergency in the declining of transmission rate coefficients. The strategies enforced during the first “state of emergency” successfully curb the development of the epidemic in the early stages, but the effective reproduction number was not maintained less than 1 after the lifting of the state of emergency.

More importantly, we emphasized the state of emergency declared for the second time recently. Based on our modelling analysis, the confirmation rates increase, and the transmission rates are smaller compared to the first declaration of state of emergency. The precision and ability of testing should have been enhanced, as put forward in the basic policies. According to the results of transmission and confirmation rates, the second nationwide declaration of state of emergency was less effective than the first time which contained the massive increment of cases within 50 days. Based on our prediction, the current state of emergency should last until May 2021 if maintaining the current strategies. It was found the isolation measures should have a greater impact on the controlling COVID-19 spreading by the comparison of various proposed combinations of strategies. Adjusting social distancing should be critical [40], which agrees with our quantitative modeling study.

The testing capacity was encouraged to be strengthened by the government basic policy and one study supported the outcome in the early spreading [38]. The confirmation rates change in this study also suggest that the testing has been improved. Among the combined strategies with different isolation and testing intensities, it could be found that overemphasizing increasing testing intensities should not be the optimal solution. After adopting stricter isolation measures, the second wave of rapid increasing infections could be controlled with moderate testing intensity. With several combinations of isolation and testing intensities, we used the model to predict *R*_*t*_ and final number of infected cases using stricter isolation measures and maintaining moderate testing intensities, and the overall infected population could decrease around 5 × 10^4^. The quantitative analysis may be able to achieve balanced control strategies to deal with the second wave of massive infections and increased untraceable cases.

The article "The Impact of the Declaration of the State of Emergency on the Spread of COVID-19: A Modeling Analysis" was published in 2021. Journal: Comput Math Methods Med.

There are several limitations in this study. This study covers a very long period of COVID-19 pandemic in Japan and assumes that people get permanently immune. Also, the application of vaccine was excluded. The production ability and the distribution should have an impact on the analysis results. Previous modeling study propose that under the scenario if *R*_*t*_ < 2.0 in Japan, herd immunity could be achieved while maintaining medical systems and lowering the severity rates [41]. Based on our analysis, the current declaration of state of emergency could result in the basic production number *R*_*t*_ around 1. If adopting the modified strategy as proposed by the modeling study, the overall infected population should be further reduced or herd immunity achieved faster with more extensive vaccination. Also, our strategies focused on the major policy change and implementation against COVID-19 in Japan. It is of more interest to evaluate the two nationwide state of emergency and propose revised containing measures for the current situation. Thus, we did not consider the regional policy change such as the declaration of the state of emergency by the Hokkaido prefecture, which may bring a small impact on the model fitting of some stages.

## Figures and Tables

**Figure 1:** The graph illustration of the SEIADR model.

**Figure 2:** The two variables representing isolation and testing intensities. Average rate of increase of untraceable cases (a). Testing index is the average testing numbers per confirmed cases per day (b).

**Figure 3:** The simulation of the early transmission stages by the model. The real accumulated confirmed cases fit well with the simulated trend (a) and locate in the 95% CI of simulated trend (b).

**Figure 4:** The fitting of confirmation rates and the testing index *χ*.

**Figure 5:** The estimation of the accumulated confirmed cases using different containing strategies in the state of emergency. Maintaining the current testing intensity with different isolating levels (a). Testing index changes to 0.8 with different isolating levels (b). Testing index changes to 1.0 with different isolating levels (c). Testing index changes to 1.2 with different isolating levels (d). Testing index changes to 1.4 with different isolating levels (e). Testing index changes to 1.6 with different isolating levels (f).

The article "The Impact of the Declaration of the State of Emergency on the Spread of COVID-19: A Modeling Analysis" was published in 2021. Journal: Comput Math Methods Med.

**Figure 6:** The contour of peak time (a) and effective reproduction number *R*_*t*_ (b) using different strategies.

**Figure 7:** Comparison between the number of forecasted cases and real cases for validation.

**Table 1:** Different stages of containing COVID-19 in Japan.

Stages	Time	Remark
1	Jan. 6 to Feb. 24 2020	Entry restrictions set for specific countries and regions [27]
2	Feb. 25 to Mar. 27 2020	Basic policy announced to containing COVID-19 spreading [26]
3	Mar. 28 to Apr. 6 2020	Basic policy modified [26]
4	Apr. 7 to Apr. 15 2020	Designated prefectures including Saitama, Chiba, Tokyo, Kanagawa, Osaka, Hyogo, and Fukuoka declared a state of emergency; the basic policies changed [26]
5	Apr. 16 to May. 24 2020	The emergency state in targeted prefectures is expanded to all 47 prefectures [26]
6	May. 25 to Jun. 24 2020	Lifting of the state of emergency [26]
7	Jun. 26 to Aug. 1 2020	Promoted strategies to support children and the elderlies [28]
8	Aug. 2 to Sep. 24 2020	Strengthened testing strategies [33]
9	Sep. 25 to Nov. 1 2020	Updated the contact conforming app [32]
10	Nov. 2 to Nov. 14 2020	Put forward COVID-19 information gathering system [31]
11	Nov. 15 to Nov. 24 2020	Provided information sharing and management support [30]
12	Nov. 25, 2020 to Jan. 7 2021	Required cooperation, preventive measures, and health management in the workplace [29]
13	Jan. 8 to Jan 27 2021	Declared another state of emergency [34]

**Table 2:** Fitted dynamic parameter values in the epidemic system.

Stages	*β*_*e*_ (per day)	*β*_*i*_ (per day)	*β*_*a*_ (per day)	*α*	*δ*	*γ*
*1*	0.1984	0.5469	0.5094	0.1590	0.1306	0.1889
*2*	0.0803	0.2454	0.2182	0.1933	0.1567	0.0565
*3*	0.3093	0.6767	0.7014	0.2581	0.4922	0.2922
*4*	0.0131	0.4395	0.3264	0.1923	0.3254	0.2211
*5*	0.0121	0.2553	0.1869	0.3340	0.1567	0.2988
*6*	0.1520	0.5290	0.4840	0.1360	0.7461	0.2000
*7*	0.1951	0.5050	0.4445	0.3293	0.4508	0.3813
*8*	0.1209	0.4499	0.4342	0.1409	0.3944	0.2977
*9*	0.1402	0.4889	0.4464	0.1211	0.5116	0.1928
*10*	0.1944	0.5425	0.5006	0.1792	0.6338	0.2186
*11*	0.1440	0.5011	0.4586	0.1248	0.6715	0.2000
*12*	0.1494	0.5183	0.4774	0.1262	0.3555	0.2388
*13*	0.0914	0.4528	0.2674	0.2915	0.5702	0.4784

## Data Availability

The data for analysis come from the following online sources: NHK: infection status in Japan, https://www3.nhk.or.jp/news/special/coronavirus/data-widget/. Tokyo metropolitan government COVID-19 information website: https://stopcovid19.metro.tokyo.lg.jp/en/cards/untracked-rate. Our World in Data: coronavirus pandemic ountry profile in Japan: https://ourworldindata.org/coronavirus/country/japan?country=∽JPN.
